The article "Vascular Endothelial Growth Factor Receptor-1 Activation Promotes Migration and Invasion of Breast Cancer Cells through Epithelial-Mesenchymal Transition" was retracted in 2022. Reasons: unreliable data; a breach of policy by an author; concerns about the data; concerns about the images.

# Vascular Endothelial Growth Factor Receptor-1 Activation Promotes Migration and Invasion of Breast Cancer Cells through Epithelial-Mesenchymal Transition

**DOI:** 10.1371/journal.pone.0065217

**Published:** 2013-06-11

**Authors:** Qian Ning, Caigang Liu, Lei Hou, Min Meng, Xiaojin Zhang, Minna Luo, Shan Shao, Xiaoxiao Zuo, Xinhan Zhao

**Affiliations:** 1 Department of Oncology, the First hospital Affiliated to School of Medicine of Xi'an Jiaotong University, Xi'an, Shaanxi Province, China; 2 Department of Oncology, First Affiliated Hospital of China Medical University, Shenyang, Liaoning Province, China; University of Nebraska Medical Center, United States of America

## Abstract

Vascular endothelial growth factor receptor-1 (VEGFR-1 or Flt-1), a tyrosine kinase receptor, is highly expressed in breast cancer tissues, but near absent in normal breast tissue. While VEGFR-1 expression is associated with poor prognosis of women with breast cancer, it is not clear whether it is involved in the aggressiveness of breast cancer. Thus, the present study examined whether VEGFR-1 activation is associated with the invasiveness of breast cancer. We reported that VEGFR-1 was detected in 60.6% of invasive breast carcinoma tissue sections. In addition, VEGFR-1 expression positively correlated with lymph node-positive tumor status, low expression level of membranous E-cadherin, and high expression levels of N-cadherin and Snail. We found that PlGF-mediated VEGFR-1 activation promoted migration and invasion in MCF-7 (luminal) cells and led to morphologic and molecular changes of epithelial-mesenchymal transition (EMT). This was blocked by the down-regulation of VEGFR-1. Conversely, down-regulation of VEGFR-1 in MDA-MB-231 (post-EMT) cells resulted in morphologic and molecular changes similar to mesenchymal-epithelial transition (MET), and exogenous PlGF could not reverse these changes. Moreover, VEGFR-1 activation led to an increase in nuclear translocation of Snail. Finally, MDA-MB-231 cells expressing shRNA against VEGFR-1 significantly decreased the tumor growth and metastasis capacity in a xenograft model. Histological examination of VEGFR-1/shRNA-expressing tumor xenografts showed up-regulation of E-cadherin and down-regulation of N-cadherin and Snail. These findings suggest that VEGFR-1 may promote breast cancer progression and metastasis, and therapies that target VEGFR-1 may be beneficial in the treatment of breast cancer patients.

## Introduction

Breast cancer is one of the most common malignant tumors in Chinese women. It's estimated that there will be more than 100 new cases per 100,000 women aged 55–69 years by 2021 [1]. Understanding the molecular mechanisms underlying the progression of breast cancer may provide ways for the development of novel antineoplastic therapies.

The article "Vascular Endothelial Growth Factor Receptor-1 Activation Promotes Migration and Invasion of Breast Cancer Cells through Epithelial-Mesenchymal Transition" was retracted in 2022. Reasons: unreliable data; a breach of policy by an author; concerns about the data; concerns about the images.

Vascular endothelial growth factor receptor-1 (VEGFR-1) is a tyrosine kinase receptor that binds vascular endothelial growth factor (VEGF)-A, VEGF-B and placental growth factor (PlGF). VEGFR-1 is the sole tyrosine kinase receptor for the later two. While VEGFR-1 is highly expressed in breast cancer tissues and breast cancer cell lines, its expression is absent or near background in normal breast tissue [2], [3]. This suggests that VEGFR-1 may play a role in tumorigenesis of breast cancer or even tumor progression and metastasis. Indeed, it has been suggested that VEGFR-1 may be an independent predicator for poor prognosis in breast carcinoma patients [4].

Epithelial-mesenchymal transition (EMT) is an essential developmental process through which cells of epithelial origin lose cell-cell contacts and cell polarity and acquire mesenchymal phenotypes, including fibroblast-like morphology with cytoskeleton reorganization, increased potential for motility, invasiveness and metastasis [5], [6]. The concept of EMT, initially developed in the field of embryology, has recently been extended to tumor invasion and metastasis. As a feature of aggressive tumors, EMT is characterized by the down-regulation of E-cadherin expression and up-regulation of N-cadherin expression [7]–[9]. Consistent with this notion, invasive ductal carcinoma exhibits a decrease in E-cadherin expression and an increase in N-cadherin expression [10], [11]. Although the role of EMT in tumor invasion and metastasis becomes a topic of interest, the molecular mechanism by which EMT is regulated has not been fully understood.

One of the key EMT regulators is Snail, which is a zinc-finger transcription factor, that represses expression of E-cadherin mRNA by binding to E-boxes in the promoter, leading to the disruption of adherin junctions (AJ) [12], [13]. Thus, Snail-deficient mouse embryos die during gastrulation due to a failure to undergo EMT [14]. The dissolution of the E-cadherin-mediated AJ is a key preliminary step in EMT. This is also the first step for tumor cells to invade surrounding tissues. Consistent with this notion, previous reports have shown that Snail mRNA is not detected in normal breast epithelium, but is expressed in 47% of infiltrating ductal breast carcinomas, and that Snail protein is over-expressed in 40.9% of invasive ductal breast carcinomas [15], [16]. It appears that the expression level of Snail is reversely correlated with E-cadherin in various carcinomas, including breast carcinoma [16].

A previous study showed that EMT resulted in an increased expression of VEGFR-1 in colonic organoids. In addition, blocking VEGFR-1 function caused massive apoptosis only in cells that underwent EMT [17]. Treatment with VEGF-A and VEGF-B, the VEGFR-1 ligands, led to morphologic and expression changes characteristic of EMT in pancreatic cells. Blocking VEGFR-1 function inhibited these changes [17], [18]. These studies demonstrated that VEGFR-1 expression or activation was associated with EMT. Since VEGFR-1 supports growth and survival of human breast carcinoma and EMT is associated with breast cancer metastasis [19]–[21], we sought to examine the association between VEGFR-1 and EMT in human breast carcinoma. In the present study, we systemically analyzed the association between clinicopathological variables with expression levels of VEGFR-1 and EMT-related proteins in 94 cases of primary invasive breast carcinoma. Finally, we demonstrated that VEGFR-1/PlGF regulated EMT in breast cancer cells *in vitro* and *in vivo*.

The article "Vascular Endothelial Growth Factor Receptor-1 Activation Promotes Migration and Invasion of Breast Cancer Cells through Epithelial-Mesenchymal Transition" was retracted in 2022. Reasons: unreliable data; a breach of policy by an author; concerns about the data; concerns about the images.

## Methods

### Cell lines, culture conditions and treatment

Human umbilical vein endothelial cells (HUVECs) and breast carcinoma cell lines (MDA-MB-453, MDA-MB-231, SK-BR-3, T-47D, BT-474 and MCF-7) were obtained from the American Type Culture Collection (ATCC, VA, USA) and cultured as instructed by ATCC [19], [22], [23]. All cells used in our experiments were at passages 3 to 15 after obtaining them from the suppliers. Cells were cultured in the absence of serum overnight prior to the treatment with PlGF (2 nmol/L, PeproTech Inc.) for the indicated periods.

### Patients and samples

We evaluated 94 invasive breast cancer samples and the matched adjacent non-cancerous samples harvested from surgical resections in the First Affiliated Hospital, College of Medicine at Jiaotong University from 2008 to 2011. All the patients (median age, 37 years; range, 21–53 years) did not receive chemotherapy, radiotherapy or hormone therapy before surgery. Their clinicopathological parameters are summarized in Table 1. Histologic types were classified according to the World Health Organization (2003). TNM staging was defined according to the American Joint Committee on Cancer (AJCC) (the 6^th^ version, 2002). All the cases were individually categorized by independent pathologists.

**Table 1:** Association analysis of clinicopathological features with expression levels of VEGFR-1, E-cadherin, N-cadherin and Snail in 94 invasive breast carcinoma samples.

Definition	VEGFR-1			E-cadherin			N-cadherin			Snail		
	Low	High	*P*	Low	High	*P*	Low	High	*P*	Low	High	*P*
Age												
<50 years	14	24	0.680	20	18	0.136	19	19	0.168	16	22	0.452
≥50 years	23	33		38	18		20	36		28	28	
Histology												
Ductal	23	41	0.321	36	28	0.112	30	34	0.122	30	34	0.985
Lobular	14	16		22	8		9	21		14	16	
Tumor size												
≤2 cm	13	18	0.938	13	18	0.022	18	13	0.007	19	12	0.029
2–5 cm	16	26		30	12		18	24		20	22	
>5 cm	8	13		15	6		3	18		5	16	
Grading												
Ι	5	5	0.569	3	7	<0.001	7	3	<0.001	9	1	0.015
ΙΙ	20	28		22	26		28	20		20	28	
ΙΙΙ	12	24		33	3		4	32		15	21	
LN status												
Negative	22	21	0.032	28	15	0.532	25	18	0.003	36	7	<0.001
Positive	15	36		30	21		14	37		8	43	
Staging												
Ι	13	16	0.072	12	17	0.001	7	22	<0.001	16	13	0.013
ΙΙ	11	30		24	17		28	13		23	18	
ΙΙΙ	13	11		22	2		4	20		5	19	
Menopausal status												
Pre-	18	26	0.773	28	16	0.717	16	28	0.344	17	27	0.136
Post-	19	31		30	20		23	27		27	23	
ER												
Negative	17	33	0.257	40	10	<0.001	15	35	0.016	10	40	<0.001
Positive	20	24		18	26		24	20		34	10	
PR												
Negative	25	27	0.054	37	15	0.036	24	28	0.307	25	27	0.784
Positive	12	30		21	21		15	27		19	23	
c-erbB-2												
0	3	17	0.09	7	13	0.088	6	14	0.418	11	9	0.546
1	13	16		19	10		14	15		16	13	
2	7	11		13	5		8	10		6	12	
3	5	7		9	3		3	9		5	7	
Not specified	9	6		10	5		8	7		6	9	
Total	37	57		58	36		39	55		44	50	

LN: lymph node; ER: estrogen receptor; PR, progesterone receptor. *P*<0.05 was considered as significant.

The article "Vascular Endothelial Growth Factor Receptor-1 Activation Promotes Migration and Invasion of Breast Cancer Cells through Epithelial-Mesenchymal Transition" was retracted in 2022. Reasons: unreliable data; a breach of policy by an author; concerns about the data; concerns about the images.

### Ethics Statement

The procedure was approved by the Committee for the Conduct of Human Ethics Committee of the First Affiliated Hospital, College of Medicine at Jiaotong University. Written informed consent was obtained from each patient enrolled in the study.

### Immunohistochemical staining

Fresh tissue specimens were fixed in 4% paraformaldehyde, embedded in paraffin, cut at 2–3 µm, and placed on slides. The slides were deparaffinized with xylene, dehydrated in graduate decreasing concentrations of ethanol, and subsequently incubated with 0.3% hydrogen peroxide for 10 min in order to block endogenous peroxidase activity. For antigen retrieval, tissue sections were heated in citrate buffer in a microwave oven followed by incubation in phosphate-buffered saline (PBS). Slides were incubated with 10% normal goat serum (in PBS) for 15 min at room temperature to block unspecific labeling and then incubated with the following primary antibodies in a humidified chamber overnight at 4°C: a rabbit polyclonal VEGFR-1 antibody (1∶50; Beijing Biosynthesis Biotechnology); a rabbit polyclonal E-cadherin antibody (1∶100; Beijing Biosynthesis Biotechnology); a rabbit polyclonal N-cadherin antibody (1∶100; Beijing Biosynthesis Biotechnology); and a rabbit polyclonal Snail antibody (1∶50; Beijing Biosynthesis Biotechnology). Following washes in PBS, sections were incubated with an appropriate secondary antibody (polymerized horseradish peroxidase [HRP]-anti rabbit IgG; Maixin-Bio, Fuzhou) for 15 min at 37°C, followed by incubation with streptavidin-peroxidase (DAKO) for 15 min at 37°C. 3,3′ -diaminobenzidine (DAB; DAKO) was applied as the chromogenic agent. Then slides were counterstained with hematoxylin, dehydrated in graded ethanol, and coverslipped. The primary antibody was replaced with PBS or normal goat serum for the blank or negative control, respectively.

The article "Vascular Endothelial Growth Factor Receptor-1 Activation Promotes Migration and Invasion of Breast Cancer Cells through Epithelial-Mesenchymal Transition" was retracted in 2022. Reasons: unreliable data; a breach of policy by an author; concerns about the data; concerns about the images.

### Immunohistochemical evaluation

The expression levels of VEGFR-1, E-cadherin, N-cadherin and Snail were independently evaluated by two investigators. Semi-quantitative analysis of staining distribution was scored as negative, +, ++, and +++ according to the percentage of cells showing immunoreactivity. Negative indicated the complete absence or weak staining in<1% of the tumor cells, + indicated focal staining in<1–10% of tumor cells, ++ indicated positive staining in 11–50% of tumor cells, and +++ indicated positive staining in>50% of tumor cells. Tumors were defined as immunopositive when>10% of tumor cells show immunoreactivity.

Expression of Snail protein was observed in the cytoplasm or nucleus or both; however, expression in only the nuclear compartment was counted as immunopositive for Snail. Expression of VEGFR-1, E-cadherin and N-cadherin were distributed in the cytoplasm and/or membrane, and both cytoplasmic and membranous expressions were considered as positive events.

### Western blotting analysis

Cells were lysed in RIPA buffer with proteinase inhibitors for 30 min on ice, and then cleared at 12,000 rpm for 20 min at 4°C. The supernatant was aliquoted for total cellular protein and its concentration was determined using the Bradford assay (Sigma

Chemicals, Bangalore, India). Nuclear extraction was performed according to the manufacturer's instructions (Pioneer Biotechnology, Inc.). Equivalent amounts of total cellular protein (10–30 µg) were subjected to reducing SDS-PAGE (8–12%) followed by blotting on a polyvinylidene difluoride (PVDF) membrane. After blocking in 5% nonfat dry milk for 2 h, membranes were incubated with the following antibodies overnight at 4°C: a rabbit monoclonal VEGFR-1 antibody (1∶10,000; Abcam); a rabbit polyclonal N-cadherin antibody (1∶800; Proteintech Group Inc.); a rabbit polyclonal vimentin antibody (1∶2,000; Proteintech Group Inc.); a rabbit polyclonal E-cadherin antibody (1∶800; Proteintech Group Inc.); a rabbit polyclonal occludin antibody (1∶1,000; Proteintech Group Inc.); a rabbit polyclonal β-catenin antibody (1∶800; Proteintech Group Inc.); a rabbit polyclonal lamin B1 antibody (1∶1,500; Proteintech Group Inc.); and a mouse monoclonal β-actin antibody (1∶1,000; Santa Cruz Biotechnology, Inc.). The membranes were then washed and incubated with a HRP-conjugated secondary antibody (Santa Cruz Biotechnology, Inc.) for 2 h at room temperature and visualized by enhanced chemiluminescence (Amersham Biosciences). Images were documented by a scanner and analyzed by Quantity One software. β-actin expression was used as a loading control for whole cell lysates, while lamin B1 expression was used as a loading control for nuclear lysates.

The article "Vascular Endothelial Growth Factor Receptor-1 Activation Promotes Migration and Invasion of Breast Cancer Cells through Epithelial-Mesenchymal Transition" was retracted in 2022. Reasons: unreliable data; a breach of policy by an author; concerns about the data; concerns about the images.

### Enzyme-linked immunoabsorbent assay (ELISA)

Breast carcinoma cells (1×10^6^) were cultured in 75 cm^2^ culture flasks containing complete medium with 10% FBS. Conditioned medium was collected on day 3 and PlGF levels were assessed using ELISA kits (R&D Systems) according to the manufacturer's instructions.

### Generation of MDA-MB-231 and MCF-7 cells stably transfected with VEGFR-1 shRNA

VEGFR-1-shRNA and control shNC in eukaryotic pGPU6/GFP/Neo plasmid vectors were obtained from Genepharma Co., Ltd (China). The target sequence for VEGFR-1-shRNA was GGACGTAACTGAAGAGGATTT as previously reported [24]. 24 h before transfection, cells were seeded onto 6-well culture plates. When cells grew to 40–70% confluence, transfection was performed using TurboFect *in vitro* Transfection Reagent (Fermentas) according to the manufacturer's instructions. 48 h post-transfection, G418 (Gibco) was added to the cell culture media at a final concentration of 500 µg/ml (MDA-MB-231) or 800 µg/ml (MCF-7) for 3 weeks. Media was changed once every 3 days. After 3 weeks, G418-resistant colonies were isolated and cultured in 96-well culture plates for further experiments.

### Cell migration and invasion assays

For *in vitro* migration assays, 24-well plates inserted with 8.0 µm pore transwells (Millipore) were utilized. 2×10^4^ cells in 200 µl of complete medium without FBS were placed on the top chamber of the insert. In the lower chamber, 500 µl of complete medium containing 10% FBS with or without PlGF was added as a chemoattractant. After 6 h (MDA-MB-231, MDA-MB-231/VEGFR-1 shRNA) or 24 h (MCF-7, MCF-7/VEGFR-1 shRNA), the cells on the top surface of the membrane were removed with a cotton swab. Migrated cells adhering to the underside of the membrane were fixed with methanol, stained with crystal violet solution and counted in 10 random fields under a microscope.

For *in vitro* invasion assays, the procedure was similar to the migration assay described above, except the membranes were coated with Matrigel and prehydrated in serum-free medium. Cells were incubated for 36 h prior to fixing and staining.

### Immunofluorescence

Cells were seeded on poly-L-lysine-coated glass coverslips in 6-well plates and received different treatments. After being fixed with 4% paraformaldehyde for 20 min, cells were permeabilized in 0.2% Triton X-100 for 10 min and blocked with normal goat serum for 30 min. Subsequently, cells were incubated with the following antibodies overnight at 4°C: a rabbit polyclonal ZO-1 antibody (1∶50 in 1%BSA; Proteintech Group Inc.); a mouse monoclonal E-cadherin antibody (1∶100 in 1%BSA; Invitrogen); a rabbit polyclonal vimentin antibody (1∶50 in 1%BSA; Proteintech Group Inc.). Slides were then washed in PBS, followed by incubation with a TRITC-conjugated secondary antibody (Wuhan Boster Biological Engineering Co., Ltd) for 2 h at room temperature. After washing in PBS, cells were incubated with DAPI (1 µg/ml, diluted in PBS) for nuclear staining for 3 min and mounted onto slides. Cells were observed under a fluorescent microscope.

The article "Vascular Endothelial Growth Factor Receptor-1 Activation Promotes Migration and Invasion of Breast Cancer Cells through Epithelial-Mesenchymal Transition" was retracted in 2022. Reasons: unreliable data; a breach of policy by an author; concerns about the data; concerns about the images.

### Tumor formation in athymic nude mice

Athymic nude mice (Silaike Laboratory Animal Co., Ltd, Shanghai, China) were used to assess the effect of VEGFR-1 shRNA on tumor growth and metastasis *in vivo*. The protocol was approved by the Animal Care and Use Committee of Xi'an Jiaotong University. Mice were divided into two groups, with six per group. Approximately 2×10^6^ cells (MDA-MB-231/shNC, MDA-MB-231/VEGFR-1 shRNA), which were suspended in 0.2 ml serum-free medium, were inoculated into the fat pad of mice. Tumor formation was measured every day. The volume of tumors was calculated using the following formula: length x width^2^×0.5. The experiments were terminated after 30 days because more than half of the mice became cachectic. Tumor-bearing athymic nude mice were observed by IVIS imaging system (IVIS spectrum, Xenogen, CA, USA) before sacrifice. The tumor tissues were removed for immunohistochemical staining.

### Statistical analysis

Statistical analysis was performed using SPSS 13.0 for Windows software (SPSS Inc., Chicago, IL). Chi-square tests and Fisher's exact tests (two-sided) were performed to assess the correlation between clinicopathological parameters and protein expression. A Spearman's rho test was used to determine the relationship among expression levels of each protein. One-way ANOVA or two-tailed Student's t-tests were used for comparisons between groups. *P*<0.05 was considered statistically significant.

## Results

### Immunohistochemical analysis of VEGFR-1, E-cadherin, N-cadherin and Snail in invasive breast carcinoma samples

We attempted to examine the expression of VEGFR-1, E-cadherin, N-cadherin and Snail in 94 invasive breast carcinoma tissues by immunohistochemistry. Association analysis between expression levels of VEGFR-1, E-cadherin, N-cadherin and Snail and clinicopathological features are summarized in Table 1. Consistent with the previous studies, VEGFR-1 protein was not detectable in normal breast tissues (Figure 1A), but was predominantly expressed in the cytoplasm of the tumor cells (Figure 1B) in 60.6% of patients (Table 1). It should be noted that both vascular endothelial cells of newly formed blood vessels and stromal cells were positive for VEGFR-1 (Figure 1B); however, only the expression of VEGFR-1 in cancer cells will be discussed in this report. VEGFR-1 expression was detected in 48.8% of samples in the lymph node-negative group and 70.6% of samples in the lymph node-positive group (Table 1). A significant association was observed between the cytoplasmic expression of VEGFR-1 and the node-positive tumor status (*P* = 0.032).

The article "Vascular Endothelial Growth Factor Receptor-1 Activation Promotes Migration and Invasion of Breast Cancer Cells through Epithelial-Mesenchymal Transition" was retracted in 2022. Reasons: unreliable data; a breach of policy by an author; concerns about the data; concerns about the images.

**Figure 1:** Immunohistochemical analysis of VEGFR-1, E-cadherin, N-cadherin and Snail in normal breast tissues and breast carcinoma tissues. VEGFR-1 (A), E-cadherin (C), N-cadherin (E), and Snail (G) expression in normal breast tissues, and VEGFR-1 (B), E-cadherin (D), N-cadherin (F) and Snail (H) expression in tumor tissues (magnification: A, E and G: 200×; B, C, D, F and H: 400×).

E-cadherin was normally present in the cell membranes of normal breast tissues, but failed to express in tumor tissues (Figure 1C and D). Approximately 61.7% (58/94) of the tumor sections showed loss or reduction of E-cadherin expression (Table 1). The reduction of E-cadherin expression was observed in 91.7% (22/24) of the late-stage and 91.7% (33/36) of the high-grade tumors, significantly more than 41.4% (12/29) of the early-stage and 30% (3/10) of the low-grade tumors (*P* = 0.001 and *P*<0.001, respectively) (Table 1). In addition, low E-cadherin expression was associated with a large tumor size and the status of estrogen receptor (ER) and progesterone receptor (PR) negativity (*P* = 0.022, *P*<0.001, and *P* = 0.036, respectively) (Table 1).

N-cadherin was absent in normal breast tissues, but highly expressed in tumor tissues (Figure 1E and F). Consistent with the association in the low-expressed E-cadherin subgroup, high N-cadherin expression was strongly associated with high-grade and late-stage tumors (*P*<0.001) (Table 1). Positive membranous N-cadherin expression also correlated with the lymph-node positive group and a negative ER status (*P* = 0.003 and *P* = 0.016, respectively) (Table 1).

Snail was not detected in normal breast tissue, but was detected in 53.2% of the tumors (Figure 1G and H and Table 1). Positive nuclear expression of Snail was associated with all adverse clinicopathologic variables, including high tumor grade, late tumor stage, lymph node positivity, and a negative ER status (Table 1). Finally, no statistically significant correlation was found between the expression levels of these four proteins and age, histology (ductal or lobular), menopausal status or the expression of c-erbB-2 (Table 1).

The article "Vascular Endothelial Growth Factor Receptor-1 Activation Promotes Migration and Invasion of Breast Cancer Cells through Epithelial-Mesenchymal Transition" was retracted in 2022. Reasons: unreliable data; a breach of policy by an author; concerns about the data; concerns about the images.

### Association between expression levels of VEGFR-1, E-cadherin, N-cadherin and Snail in invasive breast carcinoma samples

We next wanted to analyze the correlation between the expression levels of VEGFR-1 and EMT-related proteins in breast carcinoma tissues. In concordance with protein changes during EMT, high expression levels of N-cadherin and Snail were associated with weak expression of membranous E-cadherin (*P* = 0.009, r = −0.269; *P* = 0.002, r = −0.314, respectively) (Table 2). In addition, high N-cadherin expression was significantly correlated with nuclear expression of Snail (*P* = 0.016, r = 0.249) (Table 2). These analyses indicate that the invasive breast carcinoma tissues had undergone the EMT process. Surprisingly, we found that high VEGFR-1 expression was strongly associated with low E-cadherin expression (*P*<0.001, r = −0.575), high N-cadherin expression (*P*<0.001, r = 0.426), and high Snail expression (*P*<0.001, r = 0.641). These data suggest that VEGFR-1 may be involved in the regulation of EMT.

**Table 2:** Association analysis between expression levels of VEGFR-1, E-cadherin, N-cadherin and Snail in 94 invasive breast carcinoma samples.

Definition	E-cadherin			N-cadherin			Snail		
	Low	High	*P*	Low	High	*P*	Low	High	*P*
VEGFR-1									
Low	10	27	<0.001	25	12	<0.001	32	5	<0.001
High	48	9		14	43		12	45	
Spearman correlation	−0.575			0.426			0.641		
E-cadherin									
Low				18	40	0.009	20	38	0.002
High				21	15		24	12	
Spearman correlation				−0.269			−0.314		
N-cadherin									
Low							24	15	0.016
High							20	35	
Spearman correlation							0.249		

*P*<0.05 was considered statistically significant.

### Expression of VEGFR-1 and PlGF in breast cancer cell lines

To test the hypothesis that VEGFR-1 may regulate EMT in breast cancer cells, we analyzed the expression of VEGFR-1 and its corresponding ligand, PlGF, in 6 breast cancer cell lines. Both VEGFR-1 and PlGF were detected by Western blot and ELISA analyses, respectively (Figure 2A and B). We should note that there was variation of PlGF presence in the conditioned media. PlGF expression in the conditioned media of tested breast cancer cell lines was not as high as other ligands of VEGFR-1, and human PlGF was not detectable in standard culture medium containing 10% FBS (data not shown). High levels of PlGF was secreted from MDA-MB-231 but not from MCF-7 cells, while both cell lines expressed comparable levels of VEGFR-1 (Figure 2A and B). Highly tumorigenic MDA-MB-231 cells can metastasize in immunodeficient mice; however, less aggressive MCF-7 cells are only able to form tumors but not metastasize in mice [24], [25]. Therefore, we chose both MDA-MB-231 and MCF-7 cell lines for further study.

The article "Vascular Endothelial Growth Factor Receptor-1 Activation Promotes Migration and Invasion of Breast Cancer Cells through Epithelial-Mesenchymal Transition" was retracted in 2022. Reasons: unreliable data; a breach of policy by an author; concerns about the data; concerns about the images.

**Figure 2:** Analysis of VEGFR-1 and PlGF expression in human breast cancer cell lines. (A) Lysates from different breast cancer cell lines were subjected to Western blot analysis for VEGFR-1 protein expression. HUVECs were used as a positive control. β-actin is shown as a loading control. The bar graph below shows the relative protein expression levels (VEGFR-1/β-actin) among the cell lines. Data are presented as average ± s.d. from three independent experiments. *P<0.05. (B) Breast cancer cell line-derived conditioned media were subjected to ELISA for PlGF expression. Results are shown as average ± s.d. from three independent experiments. *P<0.05. Conditioned media from HUVECs were included as a positive control.

### VEGFR-1 facilitated the migration and invasion in MDA-MB-231 and MCF-7 cells

MDA-MB-231 and MCF-7 cells were stably transfected with pGPU6/GFP/Neo vectors that express shRNAs against VEGFR-1 or a control sequence (NC). Neomycin-resistant cells were characterized by Western blot using an anti-VEGFR-1 antibody. As shown in Figure 3A, VEGFR-1 protein expression was significantly decreased in MDA-MB-231 and MCF-7 cells expressing VEGFR-1-shRNA. Next, we assessed the migration and invasion capability of these cells in the presence of PlGF because it is a VEGFR-1-specific ligand [26]. PlGF treatment led to a three-fold increase in migration of MDA-MB-231 cells compared with cells without PlGF (*P*<0.05) (Figure 3B). Down-regulation of VEGFR-1 prevented PlGF-induced migration of MDA-MB-231 cells (Figure 3B). In addition, in the Matrigel-coated transwell assay in response to PlGF, the invasion of MDA-MB-231 cells increased by 1.5 fold (*P*<0.05) (Figure 3C). Reduction of VEGFR-1 expression blocked PlGF-induced invasion of MDA-MB-231 cells (Figure 3C). These findings demonstrate that the ability of MDA-MB-231 cells to migrate and invade is dependent on VEGFR-1 expression and activation. Similarly, PlGF significantly induced the migration and invasion of MCF-7 cells (Figure 3B and C). However, while migration was abrogated by down-regulating VEGFR-1, a significant decrease in invasion was not observed (Figure 3B and C).

**Figure 3:** VEGFR-1-dependent migration and invasion of MDA-MB-231 and MCF-7 cells. (A) Western blot analysis of VEGFR-1 expression in MDA-MB-231 and MCF-7 cells transfected with a shRNA against VEGFR-1. VEGFR-1 expression was significantly decreased in both MDA-MB-231 (left) and MCF-7 cells (right) expressing VEGFR-1-shRNA. The bar graph shows the relative protein expression levels among groups. β-actin was used as a loading control. Data are presented as average ± s.d. for three independent experiments. *P<0.05. (B) VEGFR-1 activation increased the migration of MDA-MB-231 and MCF-7 cells *in vitro*. PlGF induced a 3-fold increase in migration of MDA-MB-231 cells and at least a 4-fold of MCF-7 cells compared with the controls. Reduction of VEGFR-1 expression inhibited the PlGF-mediated migration of MDA-MB-231 and MCF-7 cells. (C) VEGFR-1 activation increased the invasion of MDA-MB-231 and MCF-7 cells *in vitro*. PlGF induced a 1.5-fold increase in invasion of MDA-MB-231 and 5-fold of MCF-7 cells compared with the controls. Decreased VEGFR-1 expression blocked the PlGF-mediated invasion of MDA-MB-231, but not in MCF-7 cells. Data are presented as average ± s.d. for three independent experiments. *P<0.05.

The article "Vascular Endothelial Growth Factor Receptor-1 Activation Promotes Migration and Invasion of Breast Cancer Cells through Epithelial-Mesenchymal Transition" was retracted in 2022. Reasons: unreliable data; a breach of policy by an author; concerns about the data; concerns about the images.

### VEGFR-1 activation/expression regulated EMT in MDA-MB-231 and MCF-7 cells

Surprisingly, PlGF treatment led to a spindle-shaped fibroblastic morphology in MCF-7 cells, indicating a loss of cell polarity (Figure 4A). This morphological change suggested a reminiscent of the phenotypic change of EMT. In contrast, down-regulation of VEGFR-1 resulted in MET in MDA-MB-231 cells. Post-EMT MDA-MB-231 cells lost their fibroblast-like morphology, which was accompanied by a cobblestone-like epithelial morphology (Figure 4A). ZO-1 is an important organizational component of tight junctions between epithelial cells that are the major structure in maintaining cellular polarity [27], [28]. Consistent with the phenotypic changes of losing cellular polarity, PlGF-induced VEGFR-1 activation led to a decrease in immunofluorescent staining of ZO-1 in MCF-7 cells (Figure 4B). In contrast, MDA-MB-231 cells expressing shRNA against VEGFR-1 cells acquired ZO-1 expression, indicating that the reduction of VEGFR-1 expression results in the establishment of cell polarity in post-EMT cells (Figure 4B). Approximately 40% of the MCF-7 cells underwent EMT in response to PlGF, while 30% of the MDA-MB-231 cells underwent MET due to the down-regulation of VEGFR-1 (data not shown).

**Figure 4:** VEGFR-1 expression and activation mediated EMT changes in MCF-7 and MDA-MB-231 cells. (A) PlGF treatment led to a morphological change from a cobblestone-like shape to a spindle shape in MCF-7 cells. Down-regulation of VEGFR-1 resulted in a loss of the fibroblast-like morphology in MDA-MB-231 cells. (B) Immunofluorescent analysis of ZO-1, a cell polarity protein, in MCF-7 and MDA-MB-231 cells. PlGF-activated VEGFR-1 led to a loss of cell polarity in MCF-7 cells, whereas a decrease in VEGFR-1 expression in MDA-MB-231 cells led to the re-establishment of cell polarity. (magnification 200×). (C) Immunofluorescent analysis of EMT-related regulators in MCF-7 and MDA-MB-231 cells with VEGFR-1 activation or expression. (magnification 200×). (D) Western blot analysis of mesenchymal cell markers and epithelial cell markers in MCF-7 cells when VEGFR-1 was activated by PlGF or down-regulated by shRNA. (E) Western blot analysis of mesenchymal cell markers and epithelial cell markers in MDA-MB-231 cells when VEGFR-1 was activated by PlGF or down-regulated by shRNA. β-actin was used as a loading control for whole cell lysate, while lamin B1 was used as a loading control for nuclear lysate. The bar graphs show the relative expression of proteins among each treatment groups. Data are presented as average ± s.d. for three independent experiments. *P<0.05.

The article "Vascular Endothelial Growth Factor Receptor-1 Activation Promotes Migration and Invasion of Breast Cancer Cells through Epithelial-Mesenchymal Transition" was retracted in 2022. Reasons: unreliable data; a breach of policy by an author; concerns about the data; concerns about the images.

To investigate whether the phenotypic change mediated by VEGFR-1 activation/expression was indeed EMT, we examined the expression of EMT-related regulators by immunofluorescent analysis. While MCF-7 cells normally expressed a high level of E-cadherin and an undetectable level of vimentin, PlGF-treated cells significantly reduced E-cadherin expression and increased vimentin expression. By contrast, MDA-MB-231 cells highly expressed vimentin but lacked E-cadherin expression. However, down-regulation of VEGFR-1 led to a decrease in vimentin and a concomitant increase in E-cadherin (Figure 4C). Consistently, Western blot analysis revealed that PlGF treatment led to an increase in the expression of mesenchymal cell markers and a decrease in the expression of epithelial cell markers in MCF-7 cells (Figure 4D). Furthermore, down-regulation of VEGFR-1 inhibited the PlGF-mediated expression changes (Figure 4D). Conversely, down-regulation of VEGFR-1 resulted in decreased expression levels of N-cadherin and vimentin proteins and increased expression levels of E-cadherin and occludin proteins in MDA-MB-231 cells (Figure 4E). However, PlGF treatment did not influence expression changes in these proteins (Figure 4E).

### Modulation of VEGFR-1 activation and expression led to an expression change of Snail in MDA-MB-231 and MCF-7 cells

We next investigated whether Snail, an E-cadherin repressor, was involved in VEGFR-1 activation-induced EMT. Western blot analysis showed that PlGF treatment increased Snail expression in the nucleus of MCF-7 cells (Figure 5). Consistent with our prior observations, an increase in nuclear Snail expression could be reversed by the down-regulation of VEGFR-1, even in the presence of PlGF (Figure 5). Finally, down-regulation of VEGFR-1 resulted in a decrease in nuclear Snail expression in MDA-MB-231 cells (Figure 5). However, PlGF treatment could not rescue the decreased Snail expression level mediated by VEGFR-1 down-regulation in MDA-MB-231 cells (Figure 5).

The article "Vascular Endothelial Growth Factor Receptor-1 Activation Promotes Migration and Invasion of Breast Cancer Cells through Epithelial-Mesenchymal Transition" was retracted in 2022. Reasons: unreliable data; a breach of policy by an author; concerns about the data; concerns about the images.

**Figure 5:** VEGFR-1 mediated an expression change of Snail protein in MCF-7 and MDA-MB-231 cells. Western blot analysis of Snail in nuclear extracts of MCF-7 and MDA-MB-231 cells, in which VEGFR-1 was activated by PlGF or down-regulated by shRNA. The bar graphs show the relative expression of proteins among each treatment groups. Lamin B1 was used as a loading control for nuclear lysate. Data are presented as average ± s.d. for three independent experiments. *P<0.05.

### Down-regulation of VEGFR-1 inhibited tumor metastasis in a human breast carcinoma xenograft model

Finally, we investigated the effect of down-regulation of VEGFR-1 expression on tumor growth and metastasis in female athymic nude mice. As shown in Figure 6A, tumors expressing shRNA against VEGFR-1 grew significantly slower than those in the control group (*P*<0.05). Immunohistochemical analysis showed that tumors derived from MDA-MB-231 cells expressing VEGFR-1 shRNA had an elevated level of E-cadherin, with modest levels of N-cadherin and Snail (Figure 6B). *In vivo* imaging showed that 50% (3/6) of the mice injected with MDA-MB-231/shNC had cervical metastasis, while mice treated with MDA-MB-231/VEGFR-1 shRNA did not have observable metastases (Figure 6C).

**Figure 6:** VEGFR-1 down-regulation inhibited tumor growth and metastasis in a human xenograft model. (A) Tumor-growth curve. The tumor volume in mice injected with MDA-MB-231 cells expressing VEGFR-1-shRNA was significantly smaller than the control. *P<0.05. (B) Immunohistochemical analysis of EMT related regulators in tumor sections. VEGFR-1 down-regulation in xenografts resulted in up-regulation of E-cadherin expression, with down-regulation of N-cadherin and Snail expression. (magnification: 400×). (C) *In vivo* imaging analysis. Mice treated with MDA-MB-231/shNC (a) had cervical metastasis; however, the mice treated with MDA-MB-231/VEGFR-1 shRNA (b) exhibited no observable metastasis. The reporter used GFP to show the metastasis.

## Discussion

VEGFR-1 was initially identified in vascular endothelial cells. Recently, it is apparent that VEGFR-1 is also present in several types of cancers, suggesting that VEGFR-1 plays a role in tumor invasiveness [17], [29]–[32]. However, in the literature, the percentage of positive VEGFR-1 expression in breast cancer is not consistent and its role in tumorigenesis or metastasis is not fully understood. For instance, Dale et al [33] reported that VEGFR-1 was weakly expressed in breast cancer specimens, while Schmidt et al [23] found that VEGFR-1 was expressed in 39% of breast cancer specimens, predominantly in the cytoplasm. Given that VEGFR-1 is involved in the invasiveness of other tumor types [23], [29]–[31], the purpose of the current study was to examine VEGFR-1 expression in invasive breast carcinoma samples and to examine its role in the aggressiveness of breast cancer.

The article "Vascular Endothelial Growth Factor Receptor-1 Activation Promotes Migration and Invasion of Breast Cancer Cells through Epithelial-Mesenchymal Transition" was retracted in 2022. Reasons: unreliable data; a breach of policy by an author; concerns about the data; concerns about the images.

In the present study, we found that 60.6% of the breast carcinoma tissues were positive for VEGFR-1 and that a high expression level of cytoplasmic VEGFR-1 was associated with a lymph node positive status. This is consistent with previous studies showing that VEGFR-1 expression is correlated with high metastasis and recurrence risks [33], [34]. These studies suggest that in addition to its canonical role in angiogenesis, VEGFR-1 may play a role in tumor growth and metastasis and may be an unfavorable progression indicator for patients with breast carcinoma.

EMT, a critical physiological process during development and wound healing, has been implicated in tumor progression and metastasis [35]-[39]. Through this complex process, epithelial–derived tumor cells lose intercellular tight adhesion and acquire a mesenchymal phenotype with increased migratory behavior [40]. Cadherin switching, down-regulation of epithelial cadherins (eg. E-cadherin) and up-regulation of mesenchymal cadherins (eg. N-cadherin) are necessary for increased motility and are characteristics for EMT [41]. Among the 94 breast cancer samples in our study, 61.7% showed loss or reduction of E-cadherin, while 58.5% showed positive N-cadherin expression. The correlation analysis data showed that VEGFR-1 expression was associated with low E-cadherin expression and high N-cadherin expression, suggesting that VEGFR-1 may be involved in EMT. Although VEGFR-1 activation was able to induce EMT in human pancreatic carcinoma cells [18], to our best knowledge, no studies have reported that VEGFR-1 is a possible mediator for EMT in breast cancer. In this study, since VEGFR-1 expression was strongly associated with cadherin switching during EMT, we hypothesized that VEGFR-1 could regulate EMT of breast cancer cells, leading to breast cancer progression and metastasis.

Snail-1 is a zinc-finger transcriptional factor that is overexpressed during tumor development and is associated with EMT [12], [13], [16]. We found that VEGFR-1 expression was significantly associated with Snail expression in the nucleus. This finding suggests that VEGFR-1 may regulate Snail and may result in EMT. The immuohistological data from human breast carcinoma tissues supports the hypothesis that VEGFR-1 expression may contribute to the aggressive behavior of breast cancer cells, possibly in part by mediating EMT.

The article "Vascular Endothelial Growth Factor Receptor-1 Activation Promotes Migration and Invasion of Breast Cancer Cells through Epithelial-Mesenchymal Transition" was retracted in 2022. Reasons: unreliable data; a breach of policy by an author; concerns about the data; concerns about the images.

Not only is VEGFR-1 involved in angiogenesis, it also directly contributes to tumor cell survival, and thus may attribute to the development of human breast cancer [24]. Consistent with this previous report, our data showed that all six of the breast cancer cell lines tested expressed VEGFR-1. In agreement with a prior study in which VEGF had no effect of breast cancer cell motility [3], we found that exogenous VEGF did not alter the invasion capacity of MDA-MB-231 and MCF-7 cells in the transwell assay (data not shown). Since PlGF, a ligand for VEGFR-1, acts as an autocrine factor to activate the VEGFR-1 signaling pathway [42], we detected PlGF expression in conditioned media derived from breast cancer cell lines. We found that MDA-MB-231 cells expressed a high level of PlGF, while MCF-7 cells expressed less, and this correlated with their metastatic capacity. Furthermore, we found that PlGF-mediated VEGFR-1 activation promoted the migration and invasion in breast cancer cell lines, which is consistent with the report using a pancreatic cancer model [29]. However, it remains to be elucidated how PlGF activates cytoplasmic VEGFR-1 and why VEGF does not cause activation. Consistent with these results, MDA-MB-231 breast xenografts treated with VEGFR-1/shRNA showed significant suppression of tumor growth and metastasis capacity in athymic nude mice.

Interestingly, we found that in addition to facilitating migration and invasion, VEGFR-1 activation also led to morphologic and molecular changes related to EMT. Furthermore, down-regulation of VEGFR-1 in post-EMT MDA-MB-231 cells resulted in a partial MET morphologic change, suggesting a role of VEGFR-1 in regulating EMT-MET. VEGFR-1 activation led to an increase in nuclear translocation of Snail, suggesting that VEGFR-1 activation-induced EMT might be mediated in part by Snail. Moreover, histological examination of VEGFR-1/shRNA treated tumor xenografts showed molecular changes of MET.

It has been reported that VEGFR-1 expression is significantly increased in breast cancer patients with a poor prognosis [43]. Consistent with the report, our data suggest that VEGFR-1 may be an unfavorable progression indicator for breast carcinoma patients. We provide evidence that a reduction of VEGFR-1 expression inhibits cancer cell migration and invasion *in vitro* and *in vivo*. These findings suggest that VEGFR-1 might be a potential target for neoadjuvant therapy in patients with invasive breast cancer. Specifically, our data suggests that inhibitors against intracellular VEGFR-1 may be more effective than those inhibiting extracellular VEGFR-1 because VEGFR-1 is expressed in the cytoplasm of tumor cells but not on the membrane. Furthermore, while EMT has been reported to be associated with metastasis in patients, our report is the first to suggest a possible mechanism by which VEGFR-1 may regulate EMT to promote breast cancer progression and metastasis. Therapies targeting VEGFR-1 may be a novel therapeutic approach for untreatable breast cancer patients. Additional studies are clearly needed to further understand how VEGFR-1 regulates EMT.
